The article "Intervention Effect of Rapid Rehabilitation Nursing Combined with Continuous Nursing after Discharge on Patients with Cerebral Infarction in Recovery Period and the Changes in Motor Function, Mental State, and Quality of Life" was retracted in 2023. Reasons: signs of a paper mill; compromised peer review; unreliable results or conclusions.

# Intervention Effect of Rapid Rehabilitation Nursing Combined with Continuous Nursing after Discharge on Patients with Cerebral Infarction in Recovery Period and the Changes in Motor Function, Mental State, and Quality of Life

**DOI:** 10.1155/2021/8065868

**Published:** 2021-10-15

**Authors:** Rongxiang Xie, Yi Chen, Kailang Chen, Zan Chen

**Affiliations:** ^1^Department of Rehabilitation of Traditional Chinese Medicine, Chengmai People's Hospital, Haikou, Hainan 571900, China; ^2^Department of Pediatric Urology Surgical, Xinhua Hospital Affiliated to Shanghai Jiao Tong University School of Medicine, Shanghai 200092, China; ^3^Department of Nephrology and Rheumatology, Haikou People's Hospital, Haikou, Hainan 570208, China; ^4^Department of Rehabilitation, Chengmai People's Hospital, Haikou, Hainan 571900, China

## Abstract

**Objective:**

To explore the effect of rapid rehabilitation nursing combined with continuous nursing after discharge on patients with cerebral infarction (CI) in recovery period and its influence on motor function, mental state, and quality of life.

**Methods:**

From January 2018 to December 2020, 136 patients with CI in recovery period were selected and randomly divided into control group (*n* = 68) and observation group (*n* = 68). The control group was given routine nursing, and the observation group was given rapid rehabilitation nursing combined with continuous nursing after discharge. The general clinical data of the two groups were recorded, and the nursing efficiency, modified Barthel index scale (MBI), stroke patients motor assessment scale (MAS), self-rating anxiety and depression scale (SAS and SDS), and quality of life assessment scale (QLI) were compared between the two groups.

**Results:**

The nursing effective rate of the observation group (94.12%, 64/68) was higher than that of the control group (82.35%, 56/68) (*P* < 0.05). The MBI score, MAS score, and QLI score in the observation group were higher than those in the control group, while the SAS and SDS scores in the observation group were lower than those in the control group (*P* < 0.05).

**Conclusion:**

Rapid rehabilitation nursing combined with continuous nursing after discharge can promote the rapid recovery of patients with CI in recovery period, which can improve the patient's motor function, reduce unhealthy psychology, and improve the quality of life.

## 1. Introduction

With the increasing pressure of people's life and the quickening pace of life, the incidence of cerebral infarction (CI) has been increasing in clinic, and the incidence of the population has a trend of younger age in recent years. CI refers to a disease with complete or limited brain function damage caused by acute cerebral circulation disorder, and the main symptoms of patients are limb numbness, dizziness, weakness, and other symptoms [1]. According to research reports, CI mainly occurs in middle-aged and elderly people, aged from 50 to 60 years, and the incidence rate accounts for about 25% of all cerebrovascular diseases and 70% of all stroke [2]. If CI patients are not treated effectively in time, it will affect their language and limb functions to varying degrees, and it will easily lead to paralysis, which will pose a great threat to their physical and mental health and life safety. At present, although the clinical medical technology is constantly developing, which can greatly reduce the risk of disability and death of CI patients, most CI patients still have different degrees of dysfunction after treatment and need a long time to recover, which has aroused important clinical concerns [3]. The recovery period of CI, as a transitional stage from acute stage to sequela stage, is closely related to the recovery of neurological function and prognosis of patients. Some scholars have reported that active management after CI patients are stable can reduce the risk of recurrence of CI by 90% [4]. Therefore, it is of great significance to give patients with CI scientific rehabilitation nursing during their recovery period.

Rapid rehabilitation nursing is a new nursing concept emerging in recent years. Professional nursing and rehabilitation guidance can reduce the trauma stress of patients, shorten the hospitalization time, and promote the early recovery of patients' body function [5]. Rapid rehabilitation nursing is scientific, rapid, and comprehensive, which can optimize many nursing measures during hospitalization, thus reducing stress response caused by diseases, and has played a key role in cancer, urology, and gastrointestinal and other diseases [6]. Xu's team [7] made a prospective analysis of 154 patients with colorectal cancer after operation and found that rapid rehabilitation nursing can improve patients' psychological state, complications, pain, economic pressure, and living standard.

Continuing nursing after discharge extends hospital nursing to family, which meets the nursing needs of some patients whose body function has not fully recovered after discharge. Continuing nursing after discharge can continue to implement systematic nursing for discharged patients by carrying out planned out-of-hospital guidance, which has a positive impact on improving nursing quality and improving patients' prognosis [8]. Liu's team [9] reported that the functional exercise compliance and long-term functional recovery effect of elderly hip fracture patients who have undergone continuous nursing after discharge intervention are better than those of traditional nursing patients, and they have lower adverse psychology, fewer complications, and better quality of life.

The treatment and nursing of CI have been carried out in our hospital for many years, and the medical staff in our department have many years of experience in treatment and nursing. The purpose of this study was to explore the effect of rapid rehabilitation nursing combined with continuous nursing after discharge and the changes of motor function, mental state, and quality of life of CI patients in recovery period. Specific reports are as follows.

## 2. Methods

### 2.1. Research Object

A total of 136 patients with CI in recovery period admitted to Chengmai People's Hospital from January 2018 to December 2020 were divided into a control group (*n* = 68) and an observation group (*n* = 68) by the random number table. Inclusion criteria were the following: it met the diagnostic criteria of CI [10] and was confirmed by magnetic resonance imaging or cranial CT examination; they were all in recovery period; they were aged 40–80 years; they had clear consciousness, no cognitive dysfunction, and Abbreviate Mental Test score >7 points; all patients signed informed consent. Exclusion criteria were severe mental disorder; having complete aphasia; education level below primary school; poor compliance with rehabilitation treatment; serious insufficiency of heart, liver, and kidney function; complicated with severe lung infection or pressure sore infection, severe water and electrolyte disturbance, or multiple organ dysfunction; those who have been lost to follow-up, have not received hospitalization treatment, or have withdrawn from the hospital.

### 2.2. Intervention Methods

The control group was given routine nursing and intervened for 6 months. Medical staff created a quiet and comfortable hospital environment for patients, guided them to change their unhealthy lifestyles, and maintained their mental health. Patients were instructed to strictly follow the doctor's advice and take drugs on time and in quantity and closely observed the adverse reactions after taking drugs. Family members and medical staff help patients with early daily life training, limb function recovery, balance training, walking training, etc. Before leaving the hospital, the “CI Health Knowledge Booklet” prepared by the department was distributed to the patients for reading. After discharge, the patients were instructed to take regular care and telephone follow-up.

The observation group was given rapid rehabilitation nursing combined with continuous nursing after discharge and intervened for 6 months. (1) Rapid rehabilitation nursing: ① we formed a rapid rehabilitation nursing intervention group; the team includes the leading physician, the head nurse, the responsible nurse, and the rehabilitation physician. We formulated a nursing plan according to the actual situation of patients, assisted patients to get familiar with the ward environment, explained the precautions for recovery intervention, and assisted patients to understand the relevant knowledge of CI. ② Nursing staff paid attention to psychological counseling for patients, evaluated their psychological status, actively communicated with patients, and informed them that they can recover from diseases, so as to relieve anxiety, depression, and pessimism. ③ We instructed the patient to practice sitting or supine posture and carried out swing arm rehabilitation training, so that the patient's upper limbs were brought together to his chest and gradually extend upward and unfold repeatedly. We instructed patients to carry out lower limb training and repeatedly straighten and bend back to the natural stretching part. ④ With the help of nursing staff, we carried out bed training; the training activities such as shifting, sitting up, and turning over were performed; the nurse paid attention to the patient's body posture and forbade pulling and pulling, from large joints to small joints in turn, and cooperated with appropriate massage, hot compress, and other methods to stimulate the nerve growth of patients. The degree of activity should be gradual, and the difficulty of training should be gradually increased according to the rehabilitation progress of patients. The patients' fine motor ability could be trained through activities such as calculation, looping, and pitching. ⑤ We assisted the patients in the training of balanced standing and instructed the patients to relax and keep the correct standing posture with their feet as wide as their shoulders. In the early stage, they could help with the training through ward guardrails or walking sticks. After the situation improves, they could carry out self-walking training. At the beginning of training, patients should have special personnel waiting for protection, to avoid falling, fatigue, and other phenomena. ⑥ Nurses need to set conversations that patients were interested in according to their hobbies, so as to effectively stimulate their emotions and language functions. The simple syllables, words, or paragraphs were used for training to stimulate patients to pronounce correctly and stimulate patients' hearing and language ability through books, pictures, videos, and music. (2) Continuous nursing after discharge: ① we formed a continuous nursing intervention group after discharge and formulated a nursing plan according to the actual situation of patients when they were discharged from hospital. Patients were given out-of-hospital nursing guidance by telephone or network platform, and within 1 month after the patient was discharged from the hospital, a family follow-up would be conducted every two weeks, and then a family follow-up would be conducted every other month. ② After discharge, the nursing staff actively contacted the patients or their families, inquired about their current health status in detail, evaluated their rehabilitation, strengthened their understanding of brain function rehabilitation training, and formulated detailed rehabilitation training plans, including turning over, crutches, standing, walking, eating, dressing, going to the toilet, sleeping, and functional rehabilitation training. We instructed patients' families to train patients according to the principle of strength from small to large and frequency from small to large. Because CI patients in recovery period spent a long time in bed, pressure ulcers were easy to occur, so family members needed to help patients turn over on time, and at the same time, family members needed to ensure that the bedding is clean and tidy. If family members did not remember the time and frequency of turning over, the nurse could instruct the family members to formulate a pressure sore prevention turn-over card and made a mark on the table in time after each turn-over, so as to avoid local pressure on the patient's skin. ③ The medical staff should adjust the medication scheme according to the degree of neurological impairment of patients. Medical staff gave popular science education to patients, explained the dose, frequency, and other related knowledge of drugs, informed the precautions and possible adverse reactions when taking drugs, and informed patients of the serious consequences caused by forgetting or missing drugs. ④ Medical staff gave psychological guidance to patients, increased patients' recovery confidence, introduced successful cases of rehabilitation, and explained the harm of negative psychology to them, so that patients could establish a healthy state of mind and eliminate bad emotions. If the patient's bad mood was serious, the nurse should judge whether the patient needs drug intervention according to the psychological evaluation results and clinical manifestations. ⑤ Nurses made a detailed diet structure according to the patient's condition, reasonably arranged the types of food, and guided patients to eat strictly and regularly and eat more fresh fruits and vegetables to ensure that patients had a balanced diet and adequate nutrition.

### 2.3. Observation Index

The general clinical data such as age, gender, course of disease, education level, medical expenses payment method, number of lesions, and infarction location of the two groups were recorded.

Efficacy judgment criteria: markedly effective: patients could urinate and defecate on their own, and they could basically take care of themselves in daily life; effective: patients could wear and take off their clothes by themselves, but they need help from others in getting up and walking, and their daily life was slightly affected; ineffective: the patient was still in bed, with no improvement in motor function or even worsening. Total effective rate = (markedly effective + effective)/cases × 100%.

The Modified Barthel Index (MBI) was used to evaluate patients' daily self-care ability, including 10 items such as going to the toilet, dressing, bathing, eating, and going up stairs, with a total score of 100 points. MBI score could be divided into 4 grades, and >60 points means basic self-care; 40–60 points means life needs help; 20–40 points means obvious dependence on life; <20 points means life was completely dependent. High MBI score means strong self-care ability. The retest reliability of the scale was 0.92–0.97, and the interevaluator reliability was 0.97–0.98.

The Motor Assessment Scale (MAS) was used to evaluate the motor function of patients, including 9 items, such as change of lying position, balance of sitting position, walking, upper limb function, hand movement, fine hand function, etc. A 0–6-point scoring method was used, and the ninth item was not included in the total score, only for reference, with a total score of 48 points. MAS score could be divided into 3 grades, and >33 points means mild dyskinesia; 17–32 points means moderate dyskinesia; 0–16 points means severe dyskinesia. High MAS score means good motor function. The retest reliability of the scale was 0.97, and the interevaluator reliability was 0.92.

The self-rating anxiety scale (SAS) and self-rating depression scale (SDS) were used to evaluate the mental state of patients. Both of them have 20 items and adopt 4-level scoring method. SAS score <50 points means no anxiety, 50–59 points means mild anxiety, 60–69 points means moderate anxiety, and >69 points means severe anxiety. SDS score <53 points means no depression, 53–62 points means mild depression, 63–72 points means moderate depression, and >73 points means severe depression. High scores of SAS and SDS indicate poor mental state. The retest reliability of the SAS was 0.94, and the interevaluator reliability was 0.95. The retest reliability of the SDS was 0.91, and the interevaluator reliability was 0.94.

The quality of life assessment scale (QLI) was used to evaluate patients' quality of life, including physical function, mental function, social function, and material function, with a full score of 80 points for each item. High QLI score means a good quality of life. The retest reliability of the scale was 0.79, and the interevaluator reliability was 0.81.

### 2.4. Statistical Analysis

Data were processed by the SPSS22.0, measurement data was expressed as $\bar{x}$ ± *s*, and *t*-test was used for comparison. Count data was expressed as %, and *χ*^*2*^ test was used for comparison. Differences were considered significant at *P* < 0.05.

## 3. Results

### 3.1. The General Data between the Two Groups

There were no significant differences in age, gender, course of disease, education level, medical expenses payment method, number of lesions, and infarction location of the two groups (*P* > 0.05), as illustrated in Table 1.

### 3.2. The Nursing Efficiency between the Two Groups

The nursing effective rate of the observation group (94.12%, 64/68) was higher than that of the control group (82.35%, 56/68) (*P* < 0.05), as illustrated in Table 2.

### 3.3. The Self-Care Ability between the Two Groups

After intervention, the MBI score of the observation group was higher than the control group (*P* < 0.05), as illustrated in Figure 1.

### 3.4. The Motor Function between the Two Groups

After intervention, the MAS score of the observation group was higher than the control group (*P* < 0.05), as illustrated in Figure 2.

### 3.5. The Mental State between the Two Groups

After intervention, the SAS and SDS scores of the observation group were lower than the control group (*P* < 0.05), as illustrated in Figure 3.

### 3.6. The Quality of Life between the Two Groups

After intervention, the QLI scores of the observation group were higher than the control group (*P* < 0.05), as illustrated in Figure 4.

## 4. Discussion

With the continuous progress of modern medical technology, most patients with CI can escape life-threatening after rescue. However, the neurological function of the local focus of patients with CI is deficient at the time of onset, resulting in a long recovery period after treatment. Patients often have dysfunctions in sports and cognition and other dysfunctions and cannot take care of themselves, which brings inconvenience to the daily life of patients and their families [11]. Because the structure and function of the central nervous system of CI patients have the strongest plasticity in the early stage of brain injury, and the possibility of neuron regeneration is the highest, the best time for their rehabilitation is within 6 months [12]. Therefore, the implementation of reasonable nursing measures in the early stage of CI patients' recovery will help them recover and return to society as soon as possible.

In recent years, people's living standards have been continuously improved, so people's requirements for nursing quality have also been increasing. Traditional routine intervention is single and one-sided, which can no longer meet the daily nursing needs of CI patients in recovery period. The results of this study showed that, compared with the control group, the observation group has higher nursing efficiency (94.12%) and higher MBI score and MAS score. The results showed that rapid rehabilitation nursing combined with continuous nursing after discharge was beneficial to promote the rapid rehabilitation of CI patients in recovery period and improve their motor function. We think the possible reasons are as follows: rapid rehabilitation nursing follows the principle of “people-oriented,” and by implementing a series of comprehensive nursing measures with the idea of promoting patients' rehabilitation and improving their living standards, optimizing nursing intervention programs can effectively improve patients' physiological functions and provide more scientific rehabilitation nursing for patients [13]. Some CI patients might have language barriers, so the nurses must try to mobilize the patients' desire to express themselves and stimulate their visual and linguistic nervous systems, so as to promote the recovery of their language functions. Most CI patients have varying degrees of mobility disorder, and due to the influence of nerve injury, the patient's limb control ability is significantly reduced. Under the guidance and intervention of nursing staff, rapid rehabilitation nursing helps patients build confidence in rehabilitation by actively encouraging patients to exercise themselves, and through psychological comfort, upper and lower limb massage, bed training, standing training, and other measures, the patient's nerve growth is stimulated to prevent muscle atrophy, so as to improve the self-care ability of CI patients, improve their motor function, promote the circulation of blood in their limbs, prevent the occurrence of complications, and then speed up the recovery of patients and promote them to return to normal life as soon as possible [14]. In addition, after discharge, continuing nursing belongs to the nursing visit mode of transition from hospital to society. Through various follow-up methods, continuous monitoring of discharged patients' condition, giving full professional nursing guidance to patients, and implementing individualized treatment measures can correct wrong nursing activities, solve difficulties encountered in rehabilitation training, and guide patients and their families to master basic nursing operations as much as possible, thus effectively avoiding adverse factors affecting prognosis and complications for a long time and thus improving recovery effect [15]. Medical staff timely and accurately evaluate the recovery of patients' body function during the follow-up, strengthen their families' understanding of brain function rehabilitation training, properly adjust the medication plan, implement psychological counseling for patients, introduce successful cases of rehabilitation, and provide detailed dietary guidance, thus significantly promoting the improvement of motor function, strengthening the ability of daily living, and improving the prognosis of patients with CI in recovery period [16].

Due to the inconvenience of one's own mobility, the ability to express language is significantly reduced, the emotions cannot be expressed correctly, and the recovery from the illness is relatively slow, which causes the CI patients in the recovery period to gradually lose confidence, and they are prone to anxiety, depression, depression, and other bad emotions, which seriously reduce their living standards [17]. However, because routine nursing usually stops nursing patients when they are discharged from hospital or lacks interaction with patients during follow-up, the communication between nurses and patients belongs to indoctrination education. At the same time, the nursing content of routine nursing is relatively simple, which cannot achieve targeted nursing and lacks intervention on patients' psychological status, so the patients' bad mood and quality of life have not been improved in time. Through the application of rapid rehabilitation nursing combined with continuous nursing after discharge, we found that the mental state and quality of life of the recovery period of CI patients have improved. In the process of rapid rehabilitation nursing combined with continuous nursing intervention after discharge, nurses can actively communicate with patients, do a good job of psychological counseling, evaluate patients' psychological status, explain the harm of negative psychology, and make patients realize the value and significance of continuous training for the recovery of the body, thus promoting patients' confidence in rehabilitation. Rapid rehabilitation nursing combined with continuous nursing after discharge helps patients to establish a positive attitude, helps patients master home nursing operation, promotes the integration of hospital and family, and makes patients actively cooperate with functional rehabilitation training, thus making patients physically and mentally healthy. The combined application of the two nursing modes has greatly improved patients' anxiety, depression, and other bad emotions caused by diseases, which is helpful to promote CI patients in recovery period to maintain a gradual recovery mentality, give patients great encouragement and support, and then significantly improve their living standards [18, 19].

## 5. Conclusion

Rapid rehabilitation nursing combined with continuous nursing after discharge can promote the rapid recovery of patients with CI in recovery period, which can improve the patient's motor function, reduce unhealthy psychology, and improve the quality of life. In the process of rapid rehabilitation nursing combined with continuous nursing after discharge, medical staff can formulate detailed nursing measures according to the specific situation of CI patients, which is helpful to promote patients to maintain a healthy rehabilitation mentality, has positive significance to ensure the rehabilitation effect of patients, and has clinical use and promotion value.

## Figures and Tables

**Figure 1:** The self-care ability between the two groups. *Note.* Compared with before intervention,  ^*∗*^*P* < 0.05; compared with the control group, ^#^*P* < 0.05.

**Figure 2:** The motor function between the two groups. *Note.* Compared with before intervention,  ^*∗*^*P* < 0.05; compared with the control group, ^#^*P* < 0.05.

**Figure 3:** The mental state between the two groups. *Note*. Compared with before intervention,  ^*∗*^*P* < 0.05; compared with the control group, ^#^*P* < 0.05.

**Figure 4:** The quality of life between the two groups. *Note*. Compared with before intervention,  ^*∗*^*P* < 0.05; compared with the control group, ^#^*P* < 0.05.

**Table 1:** The general data between the two groups.

General data	Control group (*n* = 68)	Observation group (*n* = 68)	*χ* ^2^ value	*P* value
Age (years, *n*, %)			0.272	0.602
40–59	30 (44.12)	27 (39.71)		
60–80	38 (55.88)	41 (60.29)		
Gender (*n*, %)			0.030	0.863
Male	36 (52.94)	37 (54.41)		
Female	32 (47.06)	31 (45.59)		
Course of disease (month, *n*, %)			0.121	0.727
1–3	39 (57.35)	41 (60.29)		
4–6	29 (42.65)	27 (39.71)		
Education level (*n*, %)			0.650	0.723
Primary school	5 (7.35)	7 (10.29)		
Junior high school	34 (50.00)	30 (44.12)		
High school or above	29 (42.65)	31 (45.59)		
Medical expenses payment method (*n*, %)			2.401	0.121
Medical insurance	59 (86.76)	52 (76.47)		
Nonmedical insurance	9 (13.24)	16 (23.53)		
Number of lesions (*n*, %)			0.641	0.726
Unilateral	17 (25.00)	14 (20.59)		
Bilateral	29 (42.65)	28 (41.18)		
Multilateral	22 (32.35)	26 (38.24)		
Infarction location (*n*, %)			0.490	0.921
Basal ganglia	24 (35.29)	25 (36.76)		
Capsula externa	7 (10.29)	5 (7.35)		
Corona radiata	20 (29.41)	19 (27.94)		
Brain lobe	17 (25.00)	19 (27.94)		

**Table 2:** The nursing efficiency between the two groups (*n*, %).

Group	Markedly effective	Effective	Ineffective	Total effective rate
Control group (*n* = 68)	35 (51.47)	21 (30.88)	12 (17.65)	56 (82.35)
Observation group (*n* = 68)	52 (76.47)	12 (17.65)	4 (5.88)	64 (94.12)
*χ* ^2^-value				4.533
*P* value				0.033

## Data Availability

The data used and/or analyzed during the current study are available from the corresponding author.
